# Clinical efficacy of posterior versus anterior instrumentation for the treatment of spinal tuberculosis in adults: a meta-analysis

This article has been retracted.

**DOI:** 10.1186/1749-799X-9-10

**Published:** 2014-02-21

**Authors:** Pinglin Yang, Xijing He, Haopeng Li, Quanjin Zang, Baohui Yang

**Affiliations:** 1 Second Department of Orthopedics, Second Affiliated Hospital of Xi’an Jiaotong University Medical School, No.157, West Fifth Road, Xi’an, Shaanxi 710004, China

**Keywords:** Adult spinal tuberculosis, Thoracic and lumbar, Meta-analysis

## Abstract

**Background:**

The aim of our study was to evaluate the clinical efficacy of posterior vs. anterior instrumentation for the treatment of spinal tuberculosis in adults.

**Methods:**

The electronic databases such as PubMed, MEDLINE, Springer, EMBASE, Google scholar, and Cochrane library were searched to select the potentially relevant reports that compared the efficacy of posterior instrumentation group (group A) with anterior instrumentation group (group B) in the treatment of spinal tuberculosis. Outcome assessments were correction of angle, loss of correction, fusion rate of the grafting bone, and complications after surgery.

**Results:**

This meta-analysis included four trials published between 2006 and 2012, involving 291 adult patients (group A, 154; group B, 137) with spinal tuberculosis. The overall meta-analysis showed that there were no significant differences (*P* > 0.01) between group A and group B in correction of angle and loss of correction at final follow-up after operation The pooled WMD (weighted mean difference) of group A and group B was 2.85 (95% CI (confidence interval) = -1.25 ~ 6.94) and 1.14 (95% CI = -3.07 ~ 5.34), respectively. Besides, no significant differences (*P* > 0.01) were observed in fusion rate of the grafting bone and complications after operation between group A and group B, and the pooled ORs (odds ratio) were 0.65 (95% CI = -0.23 ~ 1.85) and (95% CI = -0.19 ~ 1.50), respectively.

**Conclusions:**

Our results suggested that the posterior instrumentation appeared to have the same clinical outcome with the anterior instrumentation in the treatment of the adult patients with spinal tuberculosis.

## Introduction

Tuberculosis (TB) is the most common granulomatous bacterial infection in the spine [1]. Spinal tuberculosis, also called Pott's spine [2], is the most common form of extrapulmonary tuberculosis [3]. It is generally accepted that spinal TB is the most dangerous of any bone and joint TB because of its ability to cause bone destruction, deformity, and paraplegia [4]. There are conflicting guidelines and variations in clinical practice in the management of spinal tuberculosis [5]. Various modalities of treatment ranging from only antitubercular drugs to radical procedures such as anterior or combined approach surgeries have been suggested to manage spinal tuberculosis [6]. Long periods of immobilization, progressive kyphosis, and graft failure are the major postoperative problems encountered after anterior radical surgical treatment for tuberculosis of the spine [7]. Posterior fusion and instrumentation can be an effective solution for these problems [7]. Hibbs and Albee introduced posterior spinal fusion to stabilize the spine and promote healing [8,9].

Whether the clinical efficacy of posterior instrumentation for the treatment of spinal tuberculosis in adults is superior to anterior instrumentation still remains a controversy [3,10-12]. In order to achieve an integrative understanding of the clinical response of patients to posterior instrumentation (group A) and anterior instrumentation (group B), we conducted a systematic review of published findings and used meta-analysis techniques to quantitatively combine the clinic outcomes. Meta-analysis is a statistical procedure for combining the results of several studies to produce a pooled estimate of the major effect with enhanced precision [13], and it is considered a powerful tool for summarizing inconsistent results from different studies. We performed a meta-analysis to assess the correction of angle, loss of correction with final follow-up, fusion rate of the grafting bone, and complications after operation in group A and group B.

## Materials and methods

### Source of materials

The public databases including PubMed, MEDLINE and EMBASE, Springer, Elsevier Science Direct, Cochrane Library, and Google scholar were searched for relevant reports published up to December 2012. The keywords of ‘anterior,’ ‘posterior,’ ‘spinal tuberculosis,’ ‘thoracic and lumbar tuberculosis,’ ‘efficacy,’ ‘study,’ or ‘trial’ were used for searching. Meanwhile, references from retrieved papers were checked for any additional studies. We only recruited data from the fully published English paper, not from any meeting or conference abstract.

### Inclusion and exclusion criteria of the studies

The studies were included in this review if they met the following criteria: (1) prospective studies, retrospective studies, or cross-sectional studies; (2) the subjects were patients with spinal tuberculosis; (3) the studies compared the clinic outcomes of posterior instrumentation and anterior instrumentation; and (4) the studies provided odds ratio (OR) or weighted mean difference (WMD).

The studies were excluded if they met the following criteria: (1) not published in English; (2) were reviews, letters, or comments; and (3) full texts were unavailable.

### Evaluation of the quality and extraction of data

The quality of study design, sample size, and recruitment of respondents were evaluated. Initially, study titles and abstracts were read and then the full texts of potential relevant studies were screened to identify the finally eligible ones according to the inclusion criteria. Two investigators independently completed this course. Disagreements between the reviews were resolved by discussion until a consensus was reached.

We developed and modified a data extraction form after a training exercise for investigators. Data items included study details (e.g., the first author's name, year of study publication, region of participants, design of studies, etc.), characteristics of participants (e.g., age, gender, and sample size), and follow-up time with the patients. Two investigators (HL and QZ) extracted the data independently using the standard protocol, and the result was reviewed by a third investigator (BY). We contacted the authors of the studies included to obtain further information for data items that needed clarification. Discrepancies were resolved by discussion with our research team or contracting with the original investigators, who were all sent the data extraction sheets with requests for correction. We recorded the first author's name, year of publication, country, sample size, age, gender, and follow-up time with patients of group A and group B.

### Statistical analysis

The OR or WMD and their 95% confidence interval (CI) were selected as the evaluation index in current study. We assessed the within- and between-study variation or heterogeneity by testing Cochran's *Q*-statistic [14]. This heterogeneity test assessed the null hypothesis that all studies were evaluating the same effect. We also quantified the effect of heterogeneity using *I*^2^ = 100% × (*Q* - *df*)/*Q*[15], which measures the degree of inconsistency in the studies by calculating the percentage of the total variation across studies resulting from the heterogeneity rather than by chance. A significant *Q*-statistic (*P* < 0.10) or *I*^2^-statistic (*I*^2^ > 50) indicated heterogeneity across studies, and then the random effects model was used for meta-analysis. Otherwise, the fixed effects model was used. The fixed effects model assumes that all of the studies are estimating the same underlying effect and considers only within-study variation.

The overall estimate of ORs or WMD was obtained using Mantel-Haenszel method in the fixed effects model [16] and using DerSimonian and Laid method in the random effects model [17]. Pooled ORs or WMD in the meta-analysis was performed by weighting individual ORs or mean differences by the inverse of their variance. The significance of the pooled ORs or WMD was determined by the *Z*-test. Analyses were performed using the software Review Manager 5.1 (Cochrane Collaboration, http://ims.cochrane.org/revman). A *P* value less than 0.05 was considered statistically significant.

## Results

### Characteristics of eligible studies

Initially, a total of 865 papers potentially relevant to the search terms (PubMed, 232; MEDLINE, 89; Springer, 208; Elsevier Science Direct, 161; Cochrane Library, 10; Google Scholar, 165) were identified and finally only four eligible articles were included in current study. The flow chart of the study selection is shown in Figure 1. After the duplicates were removed, 238 potentially relevant studies were retained, 195 of which were excluded based on the screening of abstracts, since they were reviews (*n* = 45) not related to spinal tuberculosis (*n* = 86) or did not report posterior instrumentation (*n* = 64). The full texts of the left 43 studies were screened and 39 were excluded (16 for just only reported posterior instrumentation data but not for comparison; 23 due to no available data).

**Figure 1:** Flow diagram for selection of studies and specific reasons for exclusion from the meta-analysis.

Finally, four studies [3,10-12] were included in the meta-analysis as shown in Table 1. The eligible studies were published between 2006 and 2012 including a total of 291 spinal tuberculosis adults (group A, 154; group B, 137) who underwent the treatment with anterior or posterior instrumentation. The age of the patients ranged from 33.6 to 63.7 years old. The smallest sample size was 17 and largest was 157. The follow-up time of the included studies was from 5 to 72 months.

**Table 1:** Characteristics of studies included in the meta-analysis

**Study**	**Year of publication**	**Country**	**Sample size**	**Follow-up, mo**	**Group A**			**Group B**		
					**Sample size**	**Age in years (mean ± SD)**	**Male (%)**	**Sample size**	**Age in years (mean)**	**Male (%)**
Garg et al. [12]	2012	India	70	5 to 14	36	33.6	NA	34	34.9	NA
Lee et al. [11]	2006	Korea	17	6 to 42	10	63.70 ± 5.43	4 (40)	7	49 ± 15.87	1 (14)
Ma et al. [10]	2012	China	157	22 to 72	83	39.8 ± 1.3	32 (39)	74	38.3 ± 1.3	33 (45)
Pu et al. [3]	2012	China	47	12 to 62	25	38.1	10 (40)	22	37.8	7 (32)

*group A* posterior instrumentation group, *group B* anterior instrumentation group, *NA* not applicable.

### Overall effects of correction of angle after operation in group A vs. group B

The summary of the meta-analysis for correction of angle after operation is shown in Figure 2. The data of effect on correction of angle was available in three separate studies [3,10,12] consisting of 220 patients (group A, 117; group B, 103). The random effects model was applied to determine the correction of angle after operation between the two groups due to the evidence of heterogeneity (*Q*^2^ = 37.08, *I*^2^ = 95.0%, *P* < 0.01). The pooled WMD is 2.85 (95% CI = -1.25 ~ 6.94, *P* > 0.05) for patients in group A compared to group B, suggesting that there was no significant difference in the correction of angle after operation between these two treatment groups at the end of follow-up times.

**Figure 2:** Forest plot of correction of angle in group A vs. group B.

### Overall effects of the loss of correction with final follow-up after operation in group A vs. group B

Three separate studies [3,10,12] consisting of 220 patients (group A, 117; group B, 103) were included to assess the overall effects of the loss of correction. Heterogeneity was observed among studies (*Q*^2^ = 28.18, *I*^2^ = 93.0%, *P* < 0.01), so random effects model was applied to pool the results. No statistical significance was found in the loss of correction at final follow-up time between group A and group B (WMD = 1.14; 95% CI = -3.07 ~ 5.34, *P* > 0.05) (Figure 3).

**Figure 3:** Forest plot of loss of correction with final follow-up in group A vs. group B.

### Overall effects of fusion rate of the grafting bone after operation in group A vs. group B

The results for fusion rate of the grafting bone after operation are summarized in Figure 4. Four separate studies [3,10-12] consisting of 290 patients (group A, 153; group B, 137) were included in this meta-analysis. Testing of heterogeneity was not significant (*Q*^2^ = 0.37, *I*^2^ = 0.0%, *P* > 0.01), so fixed effects model was valid to conduct the meta-analysis. The overall meta-analysis showed that the pooled ORs were 0.65 (95% CI = -0.23 ~ 1.85, *P* > 0.05) for patients in group A compared to group B, indicating that there were no significant differences in fusion rate of the grafting bone after operation between posterior instrumentation and anterior instrumentation for the treatment of spinal tuberculosis.

**Figure 4:** Forest plot of fusion rate of the grafting bone in group A vs. group B.

### Overall effects of complications after operation in group A vs. group B

Four separate studies [3,10-12], consisting of 291 patients (group A, 154; group B, 137), were included in this meta-analysis. Because of homogeneity among the literatures (*Q*^2^ = 1.84, *I*^2^ = 0.0%, *P* > 0.01), the fixed effects model was used and postoperative complications were not found to be significantly different between group A and group B (ORs = 0.54, 95% CI = -0.19 ~ 1.50, *P* > 0.05). The result suggested that posterior instrumentation may be comparable to anterior instrumentation for the treatment of spinal tuberculosis in complications after operation (see Figure 5).

**Figure 5:** Forest plot of complication in group A vs. group B.

## Discussion

Nowadays, many studies [3,10-12] have reported clinical efficacy of posterior instrumentation group vs. anterior instrumentation group for the treatment of spinal tuberculosis in adults. But these studies have shown contradictory results due to small sample sizes or low statistical power. In our meta-analysis, we combined four studies that compared the clinical outcomes of posterior with anterior instrumentation in treatment for 291 adult patients with spinal tuberculosis. The results of this meta-analysis indicated that there were no significant differences (*P* > 0.01) in the correction of angle and loss of correction at the final follow-up time after operation between group A and group B. Besides, no significant differences (*P* > 0.01) were found in the fusion rate of the grafting bone and complications after operation between the two groups. These results demonstrated that posterior instrumentation may be equal to anterior instrumentation for the treatment of spinal tuberculosis after operation in adults.

The aims of treating spinal TB are to eradicate the infection, prevent or treat neurological deficits, correct kyphosis deformities, and finally to achieve normal sagittal contours of the spinal column, unrestricted motility, and full activities of daily living as soon as possible [1,4]. A variety of approaches are used in the surgical treatment of spinal tuberculosis, such as anterior instrumentation, posterior instrumentation, and anterior combined with posterior instrumentation. The majority of researchers favor the anterior approach due to the direct accession to the lesion, optimal visualization, and the direct and complete decompression of spinal cord provided by anterior radical surgical excision. However, the stability of anterior instrumentation appears to be a considerable issue. With the development in treating spinal tuberculosis, posterior approach has been proposed and become popular. A posterior approach in combination with internal fixation and posterior or posterolateral fusion (with or without placement of posterior interbody grafts) may be sufficient for the debridement of the infection and to allow spinal stabilization in patients with spinal tuberculous spondylitis [18]. An advantage of one-stage posterior circumferential fusion is avoiding thoracotomy and thoracoabdominal approaches, which exert considerable stress on the lungs especially so in the elderly who often suffers from impaired pulmonary function [19-21]. To date, controversy was remaining on whether anterior or posterior instrumentation should be applied in the treatment of spinal tuberculosis. In the report of Jin et al. [4], one-stage anterior interbody autografting and instrumentation were applied to treat thoracolumbar spinal tuberculosis in adults and a mean of 18° of kyphosis correction was achieved during the follow-up period. Zhao et al. [22] found that kyphotic deformity was corrected by an average of about 16° using anterior instrumentation and fusion, and in the follow-up period, correction loss was 1° (6.3%). Moon et al. [23] and Chen et al. [24], respectively, reported 44 and 29 patients with spinal TB who were treated by anterior radical surgery combined with posterior instrumentation and fusion. The average correction angle was about 18° and the loss of correction after surgery was negligible (1°–3°). It appears that anterior and posterior instrumentation can achieve similar and good results in correcting the deformity and maintaining that correction, which were in accordance with our results. However, many researchers believe that the anterior approach easily results in nerve and vascular injuries, increasing surgical complications [25,26]. In the current study, we reviewed four reports and concluded that there was no significant difference in the surgery-related complications between posterior instrumentation group and anterior instrumentation group. Therefore, further studies are needed to evaluate the complications resulted by posterior instrumentation and anterior instrumentation.

Some limitations of this study should be discussed. First of all, only published studies were included in the present meta-analysis. Thus, publication bias may have occurred and funnel plot asymmetry analysis is required. Secondly, significant heterogeneities among studies were detected in the current meta-analysis that may distort the pooled results. The degree of heterogeneity is one of the major concerns in meta-analysis for the validity of meta-analysis [27], as non-homogeneous data are liable for the misleading results. Meanwhile, different populations may lead to the heterogeneity of these trials. We should interpret these results with caution because the population from each country was not uniform. Finally, the recruited studies were not randomized controlled trial (RCT), and the numbers of studies were small (only four), so there were still need more and high-quality RCTs to test and verify the results of this meta-analysis. Therefore, we minimized the likelihood of bias by developing a detailed protocol before initiating the study, by performing a meticulous search for published studies, and using explicit methods for study selection, data extraction, and data analysis.

## Conclusions

Our results suggested that posterior instrumentation may have the same clinical outcome compared with anterior instrumentation in the treatment of spinal tuberculosis in adults.

## Abbreviations

OR: odds ratio; RCT: randomized controlled trial; TB: tuberculosis; WMD: weighted mean difference.

## Competing interests

The authors declare that they have no competing interests.

## Authors’ contributions

PY and BY participated in the design of this study, and they both performed the statistical analysis. HL carried out the study, together with QZ, and collected important background information; XH drafted the manuscript. All authors read and approved the final manuscript.
